# The Safety of Outdoor Spaces in Cold Communities Based on the Concept of Health Promotion

**DOI:** 10.1155/2022/3338210

**Published:** 2022-04-16

**Authors:** Chunyu Pang, Zhen Guan

**Affiliations:** Northeast Forestry University, Harbin 150040, China

## Abstract

With the rapid development of China's urbanization process, more and more people are pouring into cities, and this wave has inevitably caused urban housing shortages. In order to meet the living needs of citizens, a large number of communities with high housing density have emerged, resulting in many hidden safety hazards in the outdoor space of the community, forming an unhealthy community space environment. Therefore, it is imperative to build a health-promoting safety community. The thesis is aimed at studying the safety of outdoor spaces in cold communities, meeting the safety needs of community residents, and, from the evaluation of four levels of space accessibility, space identifiability, space privacy, and community service, judging the space. The main influencing factors of safety, according to the influencing factors, put forward corresponding planning strategies to provide theoretical support for the construction of safe cold community outdoor space. This paper provides a new idea for the health promotion research of community outdoor space planning, which can not only make the community outdoor environment full of sense of security but also be conducive to the sustainable development of health-promoting communities.

## 1. Introduction

The outdoor space of the cold community refers to the open-air space located between the building groups in the cold community. It has a certain purpose and communication. It is aimed at serving the residents and providing a place for the residents to communicate, watch, and relax.

Nowadays, some real estate development companies are too keen to profit from real estate and build a large number of houses, resulting in too small area of community squares and green spaces, poor lighting conditions in communities, and inability to guarantee space safety [1]. The crowded and dark living environment has a negative impact on the safe travel of residents [2]. Because of the lack of good social interaction space in many communities, the communication between residents has been significantly reduced, and the outdoor space lacks popularity, making it more difficult to achieve mutual help and love between neighbors in the traditional sense [3]. The negative impact of the community outdoor environment will destroy the quality of the community living environment [4]. In this living environment with indifferent interpersonal relationships and low security, residents are more likely to suffer from mental illnesses such as loneliness, depression, and anxiety. It can be seen that a depressing and unsafe environment will make residents lose their sense of belonging to the community [5].

These problems are common to outdoor spaces in our aging communities. However, the author conducted a survey on the communities in Harbin and other cold cities and found that the cold climate, winter snowfall, insufficient winter light, and sparse outdoor population in winter exacerbated the severity of these problems and caused great safety hazards. The crowded living environment seriously affects the development and construction of community road system, which leads to narrow road surface and poor traffic capacity, and gradually becomes potholed after a lot of traffic pressure, which reduces the safety of community traffic space. In winter, cold communities get a lot of snow, which melts on potholed roads as they heat up in the middle of the day and eventually congeals into ice. The potholed ice makes driving and residents' travel safer and prone to bloodshed. Due to the long construction time in some cold land communities, there are more illegal buildings in the community, and the community greening is unattended, which results in some problems of line of sight and blind spots in outdoor space, which ultimately leads to a decrease in the safety of outdoor space. Fewer hours of light in winter can darken already dark and crowded outdoor spaces, making them less visible, depriving residents of the ability to anticipate the safety of their outdoor spaces, increasing the likelihood of crime and accidents, and reducing the safety of their spaces. From the above, it can be concluded that there are great safety hidden dangers in outdoor space in cold communities.

The evaluation criteria of spatial health promotion include safety, satisfaction, and pleasure, of which safety is the most basic. In conclusion, in the design of outdoor space in cold communities, we should attach importance to the creation of safe space, meet the needs of different groups of people as much as possible, promote the healthy development of outdoor space in the community, and finally form a virtuous circle to create a safe outdoor space environment in the community under the concept of health promotion. Based on the concept of health promotion, this paper uses the analytic hierarchy process to establish an evaluation system for outdoor space safety in cold communities and propose space safety planning strategies, which lays a material space foundation for creating a healthy social atmosphere.

## 2. Residents' Safety Needs for Outdoor Spaces

### 2.1. Space Accessibility Requirements

Spatial accessibility refers to how easy it is to get from one point to another. Spatial accessibility reflects the degree of spatial barrier, and the lower the barrier degree, the better the accessibility [6]. The accessibility of space can measure the convenience of transportation in a space and then judge the difficulty of reaching this space.

1. Children's accessibility of outdoor activity spaces: firstly, from the analysis of children's own travel characteristics, children's physical ability and psychological development level will affect children's travel [7]. Age remains an important factor in analyzing children's range of activities. In the process of designing the outdoor activity space of the community in cold regions, the limit of physical walking distance of children and the limit of children's psychological walking distance should be taken as the starting point when formulating the space service radius; the temperature in cold regions is low in winter, and the time for children to stay outdoors is limited. The service radius of the outdoor activity space in the local community should be reasonably shortened [8, 9]
2. Elderly accessibility of outdoor activity spaces: as the age increases, the strength, agility, and control of the muscles of the elderly gradually weaken, resulting in the obstruction of motor function and the occurrence of body damage. Clinical trials have shown that the muscles of the 70-year-old will shrink in half, the exercise ability of the elderly will be weakened, and the ability to deal with unexpected situations will almost be lost. Older people's bones become brittle, and even everyday life can cause fractures [10, 11]. Therefore, the behaviors of the elderly are closely related to the barrier-free facilities. Only by building outdoor barrier-free facilities can the accessibility of the elderly in the community outdoor space be increased
3. Snow and antiskid requirements in winter: the winter climate increases the risk of accidental injury to residents. Snowfall and road icing increase the possibility of the elderly and children falling outdoors and increase the probability of residents falling and spraining in winter. Falling from a height and smashing pedestrians are always threatening the safety of pedestrians below. Therefore, in the design, attention should be paid to antiskid, snow removal, and antifreezing of outdoor roads, and the snow on eaves should be cleaned in time to reduce the impact of such factors on the safety of residents [12]

### 2.2. Space Identifiability Requirements

Residents can visually perceive the outdoor activity space and can clearly identify the path to enter the activity space, which is an important prerequisite for improving the accessibility of the community outdoor activity space. Improve the recognizability of the space, and help residents to distinguish the functions of different spaces and easily reach the activity space for outdoor activities by quickly judging the space functions. Renovating roads, boundaries, areas, nodes, and markers and setting up different places by defining boundaries, distinguishing colors and materials, etc. can effectively improve the recognition of the space.

### 2.3. Space Privacy Requirements

Safe outdoor space has a certain degree of privacy, and private outdoor space can bring residents a sense of security. The strength of privacy is mainly related to the enclosure of the side interface. Create a warm and safe space feeling through moderate enclosure, and promote the communication between neighbors.

The enclosing boundaries of communities in cold regions are mostly in the form of solid walls or fences to separate the inner and outer spaces [13]. Such boundary treatment methods are often rigid and closed. Although they isolate potential external safety hazards and facilitate community management, the rigid enclosure form cuts off the space. Extensibility results in a direct separation of space and vision. In order to ensure the privacy and vitality of the space, this paper advocates the addition of outdoor semiprivate spaces in the community.

### 2.4. Community Service Needs

1. Community mental health service needs: the fast-paced urban life has brought various pressures to community residents. Due to the lack of self-regulation ability, some residents can easily lead to emotional breakdown and then act impulsively, which not only has a negative impact on themselves but also easily affects the lives of others. Security poses a threat. Therefore, community residents' needs for mental health services should be investigated to study residents' mental health status [14]. The community needs to dispatch professional staff regularly to use psychological means to provide community residents with mental health help
2. The needs of community activities: collective activities help coordinate interpersonal relationships in the community, create a harmonious community atmosphere, and are of great significance to maintaining a safe and stable community environment

## 3. Build a Safety Evaluation System for Outdoor Spaces in Cold Communities

### 3.1. Evaluation Principles

#### 3.1.1. People-Oriented Design Principles

Starting from people's behaviors and needs and on the basis of compliance with legal norms, community members can participate in the selection process of evaluation indicators.

#### 3.1.2. Scientific Principles

The design of the outdoor space safety evaluation index system and the selection of evaluation indicators must be based on the principle of scientificity, which can objectively and truly reflect the characteristics and conditions of the internal environment of the cold community in my country and reflect the true relationship between the indicators. Each evaluation index should be typical and representative and should not be too detailed, cumbersome, or overlapping each other; it should not be too small or too simple, to avoid omission of index information, errors, and inauthenticity; index data should be easy to obtain, and the calculation method and process should be simple and easy to understand [15].

#### 3.1.3. The Principle of Typicality

The outdoor space safety evaluation index system of cold communities should be representative and should accurately reflect the comprehensive characteristics of environmental changes in cold communities in my country. Even if the number of indicators is reduced, it is necessary to facilitate data calculation and improve the reliability of results. In addition, the setting of the evaluation index system, the distribution of weights in each index, and the division of evaluation criteria should be adapted to the natural and social and economic conditions of communities in cold regions of my country.

### 3.2. Selection of Evaluation Indicators

Based on the “Healthy Community Evaluation Criteria” and guided by the concept of health promotion, this paper is aimed at meeting the safety needs of people's physical, psychological, and social adaptability. The four security elements of the community are summarized as the first-level evaluation indicators, and the four levels of spatial accessibility, spatial recognizability, spatial privacy, and community service are determined to evaluate the security of community outdoor space.

1. Evaluation indicators at the level of spatial accessibility: (1) the proportion of blind spots in space, (2) the utilization rate of outdoor fitness space, (3) the utilization rate of children's playground, (4) the utilization rate of the elderly's activity space, (5) the design and management of intelligent lighting system, (6) outdoor space lighting area, (7) road traffic system construction, (8) winter outdoor skid resistance, and (9) community trail snow volume
2. Evaluation indicators at the level of spatial recognizability: (1) community representative building ratio, (2) community characteristic landscape ratio, (3) winter ice and snow landscape ratio, and (4) IGN guidance
3. Evaluation indicators at the level of space privacy: (1) the ratio of semiprivate outdoor space and (2) the ratio of community outdoor open space
4. Evaluation indicators at the community service level:
5. Community psychological counseling: regularly provide psychological counseling to community residents and observe the mental health of community residents, which is conducive to improving the mental health of residents, alleviating incidents caused by life pressure or neighborhood conflicts, and helping to build a safe and harmonious community atmosphere
6. Participation in community activities: the degree of community residents' participation in community activities reflects the residents' sense of identity with the community, as well as the cohesion and neighborhood relationship of the community residents, to promote the residents to carry out outdoor activities and lay a good foundation for the harmonious development of the community

### 3.3. Establish an Evaluation System Framework

In this paper, the AHP is used to subdivide the outdoor space safety evaluation elements in cold communities layer by layer, which is divided into three layers: target layer, criterion layer, and index layer. To establish a hierarchical structure model, it is first necessary to conduct an in-depth analysis of the problem and then divide the factors involved into several layers according to certain principles. The selection of the indicator layer should be carried out in accordance with the principles of scientific, comprehensive, and reasonable operation. The target layers of the outdoor space safety index evaluation system in this paper are four categories: space accessibility, space identifiability, space privacy, and community service.

The following is an example of an indicator calculation process by one of the eight experts whose comments were integrated into the calculation of the weight of the indicator, so as to provide a detailed description of the process:

#### 3.3.1. Create a Hierarchical Structure

The top layer of the hierarchy is the target layer, and the evaluation index system of outdoor space safety in cold communities is presented in this paper. The guideline levels are four major community health promotion dimensions of outdoor space, namely, spatial accessibility (*A*), spatial identifiability (*B*), spatial privacy (*C*), and community service (*D*). The lowest level is the indicator layer, which is usually the specific programme or measure to achieve the goal.

#### 3.3.2. Construct a Matrix of Judgments

Compare the importance of the indicators according to the criteria in Table 1. By comparing the importance data of various indices, the conclusion of the analysis is obtained and an evaluation matrix is formed. By quantifying the judgment matrix by scalar method, the correlation between the total indicator layer and each subtarget layer, namely, *M*-*A*, *M*-*B*, *M*-*C*, and *M*-*D*, and the subtarget layer and the total indicator layer, namely, *A*‐*A*_*i*_, *B*‐*B*_*i*_, *C*‐*C*_*i*_, and *D*‐*D*_*i*_, was observed and the corresponding discriminant matrix was presented in sequence.

#### 3.3.3. Solution of Judgment Matrix

Calculation of judgment matrix is by using the integration method.

**Step 1 .**

(1) $$\begin{array}{c} M_{ij}=\frac{M_{ij}}{\sum_{i=1}^{n}M_{ij}}\left(i,j=1,2,\cdots ,n\right). \end{array}$$

In the formula, *n* is the number of evaluation indicators; *M* is the indicator set consisting of evaluation indicators; *M*_*ij*_ is *M*_*i*_ vs. *M*_*j*_ resulting in materiality.

**Step 2 .**

Add the values of each row to the normalized matrix as a benchmark

(2) $$\begin{array}{c} W_{ij}=\overset{n}{\underset{j=1}{\sum }}M_{ij}\left(i,j=1,2,\cdots ,n\right),\\ W=\left(W_{1},W_{2},W_{3},\cdots ,W_{n}\right). \end{array}$$

**Step 3 .**

Normalize processing vectors

(3) $$\begin{array}{c} W_{ij}=\frac{W_{j}}{\sum_{j=1}^{n}M_{ij}}\left(i,j=1,2,\cdots ,n\right). \end{array}$$

Calculated *W* = (*W*_1_, *W*_2_, *W*_3_, ⋯, *W*_*n*_) is the index weight vector, and the maximum characteristic root can be calculated by finally bringing in *W*.

**Step 4 .**

Test the judgment matrix for errors and perform consistency checks.

(4) $$\begin{array}{c} \text{CI}=\frac{\mu_{\max}-n}{n-1}. \end{array}$$

Of these, “*n*” represents the dimension of the matrix and “*μ*_max_” represents the maximum characteristic root of the matrix. The smaller the “CI” value, the higher the reference value of the judgment matrix.

When the satisfaction of the judgment matrix is consistent, continue to introduce the mean random concordance indicator “RI” of the judgment matrix, dividing the test value “CI” by “RI” to arrive at the test ratio:

(5) $$\begin{array}{c} \text{CR}=\frac{\text{CI}}{\text{RI}}. \end{array}$$

When “CR” is less than 0.1, the calculated index weight is valid if it passes the consistency test.

This is the basic calculation process of the weight coefficient of spatial safety evaluation index.

### 3.4. Determination of Indicator Weights

This paper uses the combination of Delphi method and analytic hierarchy process to determine the weight of the outdoor space safety evaluation index system in cold communities. First, use the Delphi method to widely solicit opinions from experts in written form, ask multiple experts to score the indicators, and establish a judgment matrix, as shown in Tables 2 and 3, for example. Then, use the analytic hierarchy process to calculate the judgment matrix for expert scoring, and finally, calculate the average value of each weight to obtain the weight value of each level of indicators, as shown in Table 4.

It can be seen from the weight factor of each index that the safety of safe community outdoor space for health promotion is most affected by the space accessibility, among which the proportion of space blind area, outdoor light environment, and road traffic safety should be considered. Secondly, when building the recognizability of outdoor space, emphasis should be placed on the recognizability of architecture, landscape, and signage. In addition, the proper creation of semiprivate spaces is also important and plays a crucial role in the privacy of outdoor spaces in communities. Finally, the community should pay some attention to the psychological counseling services for residents.

### 3.5. Evaluation Method of Space Safety

The index score is formulated on a scale of 0-5, with 5 being the highest standard. For qualitative indicators, it can be scored between 0 and 5 according to the degree of residents' emotional words. For quantitative indicators, the proportion of the indicators reaching the standard should be multiplied by the total score of 5 points to obtain the corresponding score. The calculation method of the index score of the criterion layer is to count the index scores of each subordinate index layer that belongs to the criterion layer index, multiply the corresponding score and its weight, and then add all the products to obtain the criterion layer index score.

Criterion level indicator scores are *S* = *ΣA*_*i*_∗*B*_*j*_ (*j* = 1, 2, ⋯, *n*) (where *A*_*i*_ is the index layer score and *B*_*j*_ is the corresponding weight value).

Outdoor space safety in cold communities: *N* = *ΣS*_*i*_∗*B*_*i*_ (*i* = 1, 2, 3, 4, 5) (where *S*_*i*_ is the index score value of the criterion layer and *B*_*i*_ is the corresponding weight value).

Calculate the safety of community outdoor space: the final result will be divided into 5 grades, and the scores from large to small indicate the strength of community outdoor space safety. Among them, 4-5 is the best, 3-4 is good, 2-3 is fair, 1-2 is poor, and less than 1 is the worst. Combined with the evaluation results, find out the shortcomings of community outdoor space, optimize the safety construction of community outdoor space in cold regions, guide the community outdoor space safety planning under the concept of health promotion, and lay a good foundation for the subsequent planning strategy.

## 4. Safety Planning Strategies for Outdoor Spaces in Cold Communities

### 4.1. Planning Principles

#### 4.1.1. The Principle of Fairness

The design should fully consider the special needs of the elderly, children, and other special groups for the landscape environment, provide corresponding outdoor facilities and places, and create a safe and comfortable outdoor space for all ages.

#### 4.1.2. The Principle of Suitable Climate

Cold regions have long winters and low temperatures and are vulnerable to cold winds. Therefore, the impact of cold climates should be fully considered in building layout, street design, landscape construction, and roof construction.

#### 4.1.3. Security Principle

Safety is the premise of all healthy activities, and a safe outdoor environment is the basic guarantee for leisure and social activities. In the design, we should first pay attention to resolving the elements that are not conducive to space safety, create a safe and smooth outdoor space, and build a space that can meet different groups of people: outdoor space for security needs.

#### 4.1.4. The Principle of Development

Community outdoor space planning is a long-term dynamic update process. The long-term nature of planning requires us to treat the planning with a developmental perspective, fully considering the development status of the community and the continuity of the design cycle, making it a methodological system that is constantly updated and developed, that is to say, the current space design must reserve enough for redesign: space to meet new challenges and the construction needs of the new era in the future.

### 4.2. Create a Safe Community Outdoor Space Environment

#### 4.2.1. Create a Safe Slow-Moving System for People and Vehicles to Travel Together

Roads in cold communities are an important part of the community space structure. They not only connect various groups in the community's public space and provide transportation convenience for motor vehicles and residents but also directly affect the accessibility of community spaces. In order to improve the accessibility of the space, this paper proposes the following strategies:

1. Build a road space for people and vehicles to travel together. In community planning, car dealerships and pedestrian systems should be intertwined, the focus of road design should be placed on the daily behavior of residents, the dominant position of motor vehicles should be changed, and a livable road space where people and vehicles coexist harmoniously should be formed
2. Functional compounding of road space: in addition to the basic functions of passage, the road space should have more social functions to carry residents' daily interactions and other activities. Set up functional facilities on the sidewalks on both sides of the road, such as green landscapes or rest seats, to effectively prevent the phenomenon of motor vehicles being parked indiscriminately and occupying the road. It is also possible to carry out humanized design of the ground pavement to reduce the dominance of motor vehicles through visual perception, so as to achieve the purpose of people and vehicles traveling together without affecting the daily walking life of residents
3. Optimize road network design to create a safe slow-moving environment. For communities with larger scales and relatively regular plots, a “loop + chessboard” layout can be adopted to form a safe, stable, and tidy slow-moving area. The “loop + branch” layout method limits the scope of motorized traffic activities to a certain area as much as possible, reduces the impact of motor vehicles on walking activities to the greatest extent, and creates a safe and slow path
4. Set up a corridor for the safety of the old and the young. Children and the elderly are limited by their physical abilities, so special security activity corridors should be set up for vulnerable groups such as the elderly and the young to ensure the absolute safety of slow-moving activity paths. The safe play routes for children and adolescents should be arranged according to the destination, the route to school, the route to school and the stop point, etc., and the road with fewer motor vehicles should be selected as much as possible to ensure the safety of children and adolescents during their walking process to the greatest extent. The routes for the elderly's communication activities should be arranged in combination with supermarkets, vegetable farms, parks, and other spaces, and the characteristics of the elderly to pick up and drop off children should be considered, and the routes should be appropriately arranged in combination with the children's travel routes
5. Reasonable layout of lighting facilities: (1) the lighting fixtures are suitable for combination, arrangement, shape, height, and interval. (2) The average illuminance of the Jiandao Trail is controlled at 5-10 Lx. (3) The lighting space has a sense of hierarchy, which helps to enhance the guidance of the space. (4) The style of street lamps echoes the style of community buildings. (5) Reasonably design the height of outdoor street lamps. According to the human body's demand for artificial lighting, community outdoor lamps should choose high pole lamps with a hood with a certain height. The height of the lamp should be higher than 4 m to prevent glare. (6) The illuminance of the pedestrian road lights can be placed in a lower place for lighting so that the trail is clearly visible and the illuminance is appropriate to avoid glare
6. Alleviate the security threat brought by ice and snow in the walking environment. When constructing hard paving, materials that are heat-insulating and nonslip should be selected, and the snow on the road should be cleaned in time. Reduce the possibility of the elderly and children falling due to icy roads in winter, and reduce the probability of residents falling and spraining in winter. On slopes, the antiskid strength should be increased, more antiskid materials should be selected, and handrails should be added on both sides of the road. The height of the handrails should be controlled at about 1 m, which is convenient for children to use
7. Establish a community snowfall forecasting mechanism to improve the efficiency of snow treatment. Maximize the use of snow while reducing its negative impact on the existing disaster prevention and mitigation spaces in the community, such as community roads, central green spaces, and public activity spaces, prevent snow from eroding facilities, overstocking facilities, etc. Probability of outdoor facilities to avoid bloodshed caused by collapse of heavy objects

#### 4.2.2. Enhancing Spatial Recognizability

1. Combining the existing architectural styles of the community to create a distinctive architectural layout, adding iconic buildings at the center of different organized spaces, making full use of recognizable architectural epidermis and special architectural forms to enhance residents' memory points of the space, thereby enhancing the recognizable nature of outdoor spaces
2. Give the community outdoor space different design themes in a targeted manner, such as sports and fitness, children's play, group activities, cultural exhibitions, plant viewing, and other modes, and focus on the theme in planning and design, while other function services should also be followed up, which is conducive to enhancing residents' exchanges between different community groups, enhancing the spatial characteristics and themes, and creating recognizable outdoor spaces
3. Use safe and identifiable pavement to ensure the safety of activities and increase the enthusiasm for healthy activities. Aesthetically pleasing floor coverings help to define, mark, and enhance the identity of the space, thereby increasing the enthusiasm of residents
4. Use winter snowfall to create a community-specific ice and snow landscape. Snow is used as raw material to make ice and snow sculptures; the plant conservatory irrigated by snow water and the setting of flower conservatory in winter ensure the integrity and sustainability of the outdoor landscape
5. Design of the identification system: the color, material, node environment, and surrounding landscape of the sign should maintain certain integrity. The location of the sign should be reasonable and easy to understand, and the material should be firm, corrosion-resistant, not easy to break, and easy to replace and maintain so that residents can walk more easily. Intuitive, easier to reach, and encourages more people to get involved. When setting signs, the following standards shall be followed. (1) Mileage signs, function signs, and warning signs shall be set in the community trail system. (2) The mileage and calorie signs are set every 400 m or 800 m along the route. (3) The starting point, direction, and corresponding destination are clearly marked. (4) Set up an instructive fitness guide sign every 500 m

#### 4.2.3. Soften the Enclosed Boundary of Private Space

1. Use flexible processing methods to transform the enclosed boundary. The solid wall is hollowed out, and the green landscape or microtopography is used to create a semiprivate space so that the residents have a sense of spatial domain; weaken the solidity of the enclosed boundary, and permeate the inner and outer space in terms of perception and vision, thereby increasing the boundary. The interaction of space creates a good street living environment
2. Functional renewal of community boundaries: some functions of the community's public activity space are extended to the boundary surface to become a connection between the community and the external street. After the functional renovation, the functional units such as recreation, culture, social interaction, and greening are replaced with the existing physical boundaries, which not only enhances the participation of residents but also brings new vitality to the city by utilizing the existing resources
3. Humanized design of space details: according to the functions and needs of the community space, the humanized design of the corresponding space details can not only enhance the recognizability of the community but also enhance the residents' sense of belonging to the community

#### 4.2.4. Strengthen Community Service Management

1. Provide community psychological counseling services. Increase the allocation of offline professional guidance personnel to dredge the hearts of residents. The community should incorporate the training of relevant service personnel into the routine work, systematically arrange training and advanced studies, and improve their professional knowledge and professional literacy. Give full play to the leading role of relevant personnel in promoting residents' mental health, reduce the probability that residents often quarrel with their neighbors due to emotional pressure, and help create a safe and harmonious social atmosphere
2. Organize community-wide outdoor activities on time. Under the guidance of the community, community residents spontaneously organize different activity groups and give full play to the organizational role of residents with strong organization or professional expertise. The community should use part of the planning special funds to provide support to residents and help them carry out corresponding activities, which not only gives full play to the enthusiasm of residents, attracts more residents to participate in activities, enhances emotional communication between community neighbors, and promotes community managers and community residents. The beneficial exchanges will help to create a safe and harmonious community atmosphere and reduce the occurrence of community conflicts

## 5. Conclusion

This article seeks to explore safety standards for health-promoting communities. This paper analyzes the safety needs of residents in cold regions, constructs an evaluation system for outdoor spaces in cold regions by analyzing the factors affecting the safety of outdoor spaces, and proposes outdoor space safety planning strategies, which brings new blood into the community planning work. Suggestions are provided for the construction of community outdoor space safety.

## Figures and Tables

**Table 1:** Meaning of indicator importance scale.

Importance scale	Meaning
1	Metric *i* and metric *j* are equally important
3	Metric *i* is slightly more important than metric *j*
5	Metric *i* is significantly more important than metric *j*
7	Metric *i* is strongly more important than metric *j*
9	Metric *i* is extremely important than metric *j*
2, 4, 6, 8	The importance is between 1, 3, 5, 7, and 9
Reciprocal	Inverse comparison between two factors

Source of the chart: the author's own drawing.

**Table 2:** *M* judgment matrix and index weight of outdoor space safety evaluation system in cold communities.

*M*	*A*	*B*	*C*	*D*	Weight factor
*A*	1	2	2	3	0.4249
*B*	1/2	1	2	2	0.2701
*C*	1/2	1/2	1	1	0.1613
*D*	1/3	1/2	1	1	0.1438

Source of the chart: the author's own drawing.

**Table 3:** Spatial accessibility index *A*-*A*_*j*_ judgment matrix and index weight.

*A*	*A*1	*A*2	*A*3	*A*4	*A*5	*A*6	*A*7	*A*8	*A*9	Weight factor
*A*1	1	2	2	2	1	1/2	1	1	2	0.0518
*A*2	1/2	1	1	1	1/2	1/3	1/2	1/2	1	0.0268
*A*3	1/2	1	1	1	1/2	1/3	1/2	1/2	2	0.0295
*A*4	1/2	1	1	1	1	1/3	1/3	1/3	1	0.0276
*A*5	1	2	2	1	1	1/2	1/2	2	3	0.0529
*A*6	2	3	3	3	2	1	3	2	3	0.0989
*A*7	1	2	2	3	2	1/3	1	2	3	0.0662
*A*8	1	2	2	3	1/2	1/2	1/2	1	1	0.0456
*A*9	1/2	1	1/2	1	1/3	1/3	1/3	1	1	0.0255

Source of the chart: the author's own drawing.

**Table 4:** Weights of evaluation indicators for outdoor space safety in cold communities under the concept of health promotion.

Target layer	Criterion layer	Indicator layer	Weight factor	Indicator layer
*M*: cold area community outdoor space safety evaluation system	*A*: spatial accessibility metrics	0.4249	*A*1: the proportion of space blind spots	0.0518
			*A*2: outdoor fitness space utilization	0.0268
			*A*3: utilization of children's playground	0.0295
			*A*4: utilization of venues for seniors	0.0276
			*A*5: intelligent lighting system design and management	0.0529
			*A*6: outdoor space lighting area	0.0989
			*A*7: construction of road traffic system	0.0662
			*A*8: antiskid degree of outdoor in winter	0.0456
			*A*9: community trail snow coverage	0.0255
	*B*: spatial identifiability metrics	0.2701	*B*1: the proportion of representative buildings in the community	0.0962
			*B*2: community characteristic landscape ratio	0.0796
			*B*3: winter ice and snow landscape ratio	0.0265
			*B*4: logo guide	0.0677
	*C*: spatial privacy indicators	0.1613	*C*1: semiprivate outdoor space ratio	0.1210
			*C*2: community outdoor open space ratio	0.0403
	*D*: community service indicators	0.1438	*D*1: community psychological counseling	0.0359
			*D*2: participation in community activities	0.1078

Source: author's own drawing.

## Data Availability

The data used to support the findings of this study are available from the corresponding author upon request.
